# Clinical Effect of Catgut Embedding plus Warm Needle Moxibustion on Improving Inflammation and Quality of Life of Knee Osteoarthritis Patients

**DOI:** 10.1155/2022/5315619

**Published:** 2022-10-05

**Authors:** Di Zhang, Shuanglin Song, Zhenyu Bian, Zhen Huang

**Affiliations:** Department of Acupuncture and Massage, Affiliated Hangzhou First People's Hospital, Zhejiang University School of Medicine, Hangzhou, Zhejiang 310006, China

## Abstract

**Objective:**

To clarify influence of catgut embedding plus warm needle moxibustion on improving inflammation and quality of life of knee osteoarthritis patients.

**Materials and Methods:**

The data of 120 patients with knee osteoarthritis admitted to our hospital from June 2018 to June 2021 were used for retrospective analysis. Patients were divided into control group and observation group in a random manner, with 60 cases each. The control group was orally administrated with one diclofenac sodium sustained-release tablet (100 mg) once a day, for 8 courses with 7 days for each course. The observation group underwent catgut embedding plus warm needle moxibustion.

**Results:**

The Western Ontario and McMaster Universities Arthritis Index and gonitis Lequesne scores in two groups were decreased after treatment and were lower in observation group than control group (*P* < 0.05). Quality of life scores presented elevation after treatment and were higher in observation group than control group (*P* < 0.05). Curative efficacy presented no difference between two groups (*P* > 0.05), while clinical cure rate was higher in observation group than control group (*X*2 = 8.257, *P* = 0.006).

**Conclusion:**

Warm needle moxibustion plus functional exercise can effectively improve clinical symptoms of knee osteoarthritis patients, and improve their knee joint function and inflammatory response.

## 1. Introduction

Knee osteoarthritis (KOA) is a degenerative disease characterized by knee cartilage degeneration and reactive hyperplasia [1], which is more common in the elderly. Because the main clinical manifestations of this disease are knee joint swelling and pain as well as deformity, which reduces quality of life of patients, brings serious pain and economic burden to patients, and what kind of treatment methods should be adopted to alleviate clinical symptoms and delay disease progression has become a current problem that needs to be solved urgently [2]. At present, the treatment of KOA in modern medicine is mainly based on physical, drug, and surgical therapies. Physical therapy includes heat compress, electrotherapy, wax therapy, and other treatment methods [3]. Drug therapy mostly uses nonsteroidal anti-inflammatory drugs (NSAIDs), analgesics, knee joint drug injection, etc. to achieve the therapeutic effect of pain relief, anti-inflammation, and improvement of knee joint function, but drug therapy has certain side effects, thus it is not suitable for long-term use. Surgical therapy for KOA includes arthroscopy, osteotomy, and joint replacement [4, 5], which can effectively improve symptoms, but patients are quite afraid and need to face higher surgical risks and anesthesia risks when undergoing surgical therapy, especially in patients with severe underlying diseases.

In traditional Chinese medicine (TCM), KOA belongs to the category of “rheumatism”, which is recorded in the *Inner Canon of Huangdi*. The TCM believes that this disease is mostly caused by liver and kidney deficiency, invasion by external pathogens, and consumptive wear and tear. The main treatment methods of TCM for this disease include oral administration, external application, fumigation, acupuncture, and massage. Each treatment method can be used alone or cooperated with each other to reduce swelling, relieve pain, and improve joint function. Furthermore, TCM treatment has the advantages of convenience, less side effects, easy promotion, relatively small economic burden, etc., and is easily accepted by patients [6]. Acupoint catgut embedding belongs to a traditional external therapy in China, which is an extension and development of acupuncture and moxibustion therapy. According to the guidance of meridians theory, intestinal suture or absorbable surgical suture is implanted into corresponding acupoints, and the decomposition and absorption process can produce long-lasting, slow, and stable acupuncture and moxibustion effects at acupoints. At present, it has been widely applied in treating migraine, sciatica, low back pain, and other acute and chronic pain, with certain efficacy, low cost and low adverse reactions [7]. Catgut embedding therapy combines traditional needle-knife therapy with acupoint catgut embedding therapy, making full use of needle-knife to precisely release the adhesion tissue, scars, and contractures around the knee joint, and acupoint catgut embedding to continuously stimulate the surrounding tissue, in order to facilitate local blood circulation, improve knee joint function, relieve pain, delay disease progression, and improve quality of life of patients [8].

In our research, we aimed to investigate the efficacy of catgut embedding combined with warm needle moxibustion on KOA, and to clarify its impact on quality of life of patients.

## 2. Materials and Methods

### 2.1. General Data

The data of 120 patients with KOA admitted to our hospital from June 2018 to June 2021 were chosen for retrospective analysis and divided into two groups in a random manner. There were 60 cases in control group, including 32 males and 28 females; the age was 41-70 years, average: 59.52 ± 9.45 years, the disease duration was 0.5-10 years, average: 5.57 ± 1.38 years. There were 60 cases in observation group, including 34 males and 26 females; the age was 40-69 years, average: 58.05 ± 9.12 years, the disease duration was 0.5-10 years, average: 5.65 ± 1.42 years. Inclusion criteria: (1) meet the relevant diagnostic criteria in the *Guidelines for the Diagnosis and Treatment of Osteoarthritis (2017 version)*; (2) KOA grade: II-IV; (3) those who did not receive other treatments within 1 month. Exclusion criteria: (1) those complicated with severe cardiovascular and cerebrovascular, liver, and renal system diseases; (2) those complicated with rheumatoid arthritis, septic arthritis, meniscus injury, joint tuberculosis, and other knee joint diseases; (3) those with blood diseases, mental disorders, and malignant tumors; (4) those with allergic constitution. Age, disease duration, KOA grade, and other data of KOA patients presented no difference but balance between two groups (*P* > 0.05). This study was approved by the Ethics Committee of Affiliated Hangzhou First People's Hospital, Zhejiang University School of Medicine, and all patients signed informed consent.

### 2.2. Treatment Methods

The control group was administrated conventional nonsteroidal anti-inflammatory drugs [9], and our hospital administrated diclofenac sodium sustained-release tablets to patients, 1 tablet (100 mg) orally once a day, 7 days as a course of treatment, with continuous treatment for 8 courses.

The observation group underwent catgut embedding plus warm needle moxibustion therapy. The patients were given warm needle moxibustion and acupoints such as the inner and outer knee eyes, Yanglingquan, Yinlingquan, Liangqiu, and Zusanli were chosen on the affected side. Routine disinfection of the skin, oblique puncturing of the inner and outer knees and inwards, straight puncturing in Yanglingquan, Yinlingquan, Liangqiu, and Zusanli, retention of the needles for 30 min after obtaining Qi, moxibustion in Liangqiu and Zusanli for 2 puncture/time, 1 time/d. Catgut embedding acupoints: Xuehai, Liangqiu, Yanglingquan, Ashi, popliteus point, and goose foot point. The patients took the supine position, with the knee joint fully exposed, the joint was flexed 30°-45°, and the back of the knee joint was bolstered. The operator stood on the affected side, operated in strict accordance with the surgical aseptic principle, and disinfected the skin with an iodophor cotton ball, and the disinfection area was supposed to include a range of 10 cm around the acupoint. The skin was disinfected from the acupoints to the peripheral skin three times in total, and then wiped with an alcohol cotton ball to remove the iodine on the skin surface. The catgut embedding needle-knife was taken out, the polyglycolide absorbable thread package (PGLA, catgut length: 1.5 cm) was opened with sterile scissors, the operator wore sterile gloves, and gently pulled the needle core handle of catgut embedding needle-knife back. The absorbable catgut was taken out with sterile tweezers, the catgut embedding needle-knife was inserted with a length of 0.75 cm, and the catgut was bent into a V shape. The thumb of the left hand was used to determine the acupoint again, the index finger and middle finger of the left hand were used to tighten the skin around the acupoint, and the catgut embedding needle-knife was pressed against the skin of the acupoint with the right hand. The direction of the blade was parallel to the longitudinal axis of the lower limb. After quickly piercing the skin, the needle was inserted slowly, with depth of 1.5 cm (based on the scale of the needle) and avoided entering the joint cavity. The needle knife was used to cut the local tissue longitudinally and rotated several times. When the needle felt loose, the needle handle was pushed down, the catgut was buried into the acupoint, the needle was slowly pulled out, and the acupoint was pressed at the same time. When there was no blood oozing out of the skin, the same method was used to puncture other acupoints on the front of the knee joint, and a sterile patch was applied after the puncture was completed. The patients were changed to the prone position to fully expose the acupoints behind the knee joint. After the operator changed sterile gloves, the same method was used to sterilize acupuncture at a fixed point. After the operation, the dressing was changed once a day for the first three days, and then every two days to avoid infection, once every 2 weeks, 4 weeks as a course of treatment, with continuous treatment for 2 courses. The patients in both groups were given standardized health guidance and performed functional exercises of the knee joint.

### 2.3. Adverse Events

Adverse events were defined as unanticipated and unanticipated signs, symptoms, and diseases that occurred after treatment during the course of this clinical study and were not necessarily caused by this clinical study. Subjects were suspended from trial treatment if a serious adverse event (SAE) occurred during the course of the study, and their participation was discontinued if continued treatment was considered dangerous to the subject and the adverse event was related to the intervention.

### 2.4. Withdrawal and Dropout

All participants had the right to withdraw from the study at any time. If the subject refuses to continue, withdraws consent, or violates inclusion or exclusion criteria, participation will end at any stage. In addition, the investigators recorded the completion of the study and the reasons for stopping the trial.

### 2.5. Observation Indicators

1. The KOS self-assessment scale was used to evaluate the condition. The Western Ontario and McMaster Universities (WOMAC) Osteoarthritis Index mainly evaluated from three aspects: pain degree, stiffness degree, and difficulty in performing daily activities [10]. It included 24 basic symptoms and signs of osteoarthritis. The total score ranged 0-96 points. The index measures 2 questions for stiffness degree (score range 0–8), 5 questions for pain degree (score range 0–20), and 17 questions for difficulty in performing daily activities (score range 0–68). The higher score suggested the more serious disease. Each of the 24 items was divided into 3 grades: asymptomatic 0, mild 1, moderate 2, severe 3, and extreme 4
2. Lequesne score for osteoarthritis [11] was mainly used to evaluate knee joint function and disease progression. It consisted of three parts: knee joint pain score, walking distance score, and daily living disorder score. The score ranged 0-24 points. A high score indicated a severe degree of knee osteoarthritis and poor knee function
3. MMP-3, MMP-9, interleukin-1 (IL-1), and tumor necrosis factor-*α* (TNF-*α*) levels in two groups before treatment, and after 2 courses of treatment were assessed by ELISA kit (Thermo Fisher, USA)
4. The health survey short-form MOS SF-36 evaluated quality of life [12], including 8 dimensions of Physiological Functioning (PF), Role-Physical (RP), Bodily Pain (BP), General Health (GH), Vitality (VT), Social Functioning (SF), Role-Emotional (RE), and Mental Health (MH), total 36 items, and each item was scored on a 0-100 range, the conversion score was calculated using the standard formula: [original score − lowest possible score)/possible score range ×100%], by percentage scale. The higher score suggested the better quality of life
5. Referring to the *Efficacy Criteria for Diagnosis of Diseases in Traditional Chinese Medicine*, clinical efficacy was classified into 4 grades: clinical cure (symptoms disappeared, functional activity returned to normal, and erythrocyte sedimentation rate, rheumatoid factor, immunoglobulin, and other related laboratory indicators, as well as X-ray and other physical and chemical test results were normal), markedly effective (symptoms, functional activities, laboratory indicators, X-ray, and other physical and chemical test results were remarkably improved, but did not reach the clinical cure standard), improved (symptoms, functional activities, laboratory indicators, X-ray, and other physical and chemical test results were improved, but not remarkably, not reaching the markedly effective standard), and ineffective (symptoms, functional activities, laboratory indicators, X-ray, and other physical and chemical examination results did not improve or even worsened)

### 2.6. Statistical Analysis

SPSS 20.0 software was used for data analysis. Measurement data were expressed as (*x* ± *s*), independent samples *t*-test was used for comparison between groups, and paired sample *t*-test was used for both within groups. Enumeration data were expressed as rate (%), and *x*^2^ test was used for comparison between groups. *P* < 0.05 meant there was statistical significance.

## 3. Results

### 3.1. Comparison of WOMAC Scores and Total Scores of Pain, Stiffness, and Daily Activity Difficulty between Two Groups before and after Treatment

WOMAC scores and total scores presented no difference between two groups before treatment (*P* > 0.05). WOMAC scores and total scores in two groups after treatment presented depletion relative to those before treatment, with statistical significance (*P* < 0.05). WOMAC scores and total scores in treatment group presented depletion relative to control group after treatment, with statistical significance (*P* < 0.05, Figure 1).

### 3.2. Comparison of Inflammatory Cytokine Levels between Two Groups before and after Treatment

Serum MMP-3, MMP-9, IL-1, and TNF-*α* levels presented no difference between control group and observation group before treatment (*P* > 0.05). Relative to control group, serum MMP-3, MMP-9, IL-1, and TNF-*α* levels in observation group presented depletion after 1 month of treatment (*P* < 0.05, Figure 2).

### 3.3. Comparison of Quality of Life between Two Groups before and after Treatment

Quality of life scores of each dimension and total scores presented no difference between two groups before treatment (*P* > 0.05). After treatment, quality of life scores of each dimension and total scores presented elevation relative to those before treatment, and observation group presented elevation relative to control group, with statistical significance (*P* < 0.05, Figure 3).

### 3.4. Comparison of Lequesne Scores for Osteoarthritis between Two Groups before and after Treatment

After comparative analysis, gonitis Lequesne scores presented no difference in two groups before treatment (*P* > 0.05), which was comparable. Gonitis Lequesne scores in two groups after treatment presented depletion relative to those before treatment, with statistical significance (*P* < 0.001). Gonitis Lequesne scores in observation group presented depletion relative to control group, with statistical significance (*P* < 0.05, Table 1).

### 3.5. Comparison of Clinical Efficacy between Two Groups

Curative efficacy presented no difference between two groups (*P* > 0.05), but clinical cure rate in observation group presented elevation relative to control group, with statistical significance (*x*^2^ = 8.257, *P* = 0.006, Table 2).

## 4. Discussion

KOA, also known as proliferative arthritis, is the most common chronic disease among knee joint diseases. The pathogenesis of KOA is still unclear in modern medicine [1, 13, 14]. There are more women than men in KOA patients, the age of onset is more than 40 years old, and most of them are obese people. The incidence is mostly due to the disorder of limb alignment and the release of inflammatory mediators caused by various factors such as age, weight, and trauma. Modern medical treatment of KOA includes drug therapy and surgical treatment. Drug therapy includes NSAIDs, analgesics, and intra-articular injection, and NSAIDs is widely used and has good anti-inflammatory and analgesic effects, but it may increase bleeding tendency and cause liver, kidney, and gastrointestinal damage during use.

Catgut embedding plus warm needle moxibustion is a new treatment method developed from traditional acupuncture and acupoint thread embedding. *Miraculous Pivot·Nine Needles and Twelve Source Acupoints* pointed out: “A sharp needle, with a blade on three sides, can be used to treat stubborn old diseases,…. Long needles, sharp, and slender, can be used to treat long-standing paralysis”. *Miraculous Pivot·Needles* pointed out: “Nine (big) needles are used to clear the nine orifices and remove the evil energy between the three hundred and sixty-five festivals in the whole body. This is called different needles have different functions and indications.” It is suggested that the use of acupuncture to release and decompress the soft tissues such as joint capsule and fascia of the whole body can achieve the purpose of curing pain with looseness. Acupuncture can release scars and soft tissue adhesions, protect articular cartilage cells, and maintain mechanical balance, which is a commonly used clinical treatment method [15, 16]. The acupoint catgut embedding 100 is to embed catgut or surgical absorbable thread into the treatment acupoint, and use the thread to continuously stimulate the acupoint to achieve the therapeutic function. *Miraculous Pivot: Beginning and End* pointed out: “Those who have been ill for a long time will have deep penetration of pathogens. For such chronic diseases, deep acupuncture is required, and the needles are kept for a long time.” Acupoint catgut embedding can achieve continuous stimulation locally, and at the same time, it reduces the possible adverse reactions of long-term acupuncture to local tissues, and has the characteristics of “replacing the thread with needles.” Catgut embedding plus warm needle moxibustion combines traditional acupuncture and acupoint thread embedding, and has both the relaxing effect of traditional warm needle moxibustion and the continuous stimulation of acupoint thread embedding. The therapeutic effect is better than that of warm needle moxibustion or acupoint catgut embedding alone. Relative to warm needle moxibustion, it has the advantages of high stimulation intensity and long duration of curative efficacy. Our research will provide a clinical basis for exploring the effectiveness of catgut embedding plus warm needle moxibustion by observing the efficacy of catgut embedding plus warm needle moxibustion on KOA.

The WOMAC scores can effectively reflect the patient's condition before and after treatment, such as the patient's satisfaction. It has a high reliability in the assessment of KOA [17]. Herein, WOMAC scores in treatment group by catgut embedding plus warm needle moxibustion presented depletion relative to control group, suggesting that warm needle moxibustion for KOA can improve clinical symptoms and relieve stiffness and pain symptoms, and joint function is better restored.

Inflammatory cytokines exert a vital role in KOA occurrence and development. Inflammatory cytokines stimulate synovial cells to secrete massive IL-1, promote the synthesis of MMP-3, and MMP-9, and further degrade articular cartilage, affecting bone metabolism [18]. TNF-*α* can promote the formation of new blood vessels in the synovium, elevate the permeability of vascular wall, and aggravate inflammatory response of joints. Angiopoietin I can promote angiogenesis and stimulate synovial and cartilage lesions [19]. The elevated serum levels of MMP-3, MMP-9, IL-1, and TNF-*α* indicate that patients' bone and cartilage structures are being destroyed. Herein, after 1 month of treatment, relative to control group, serum MMP-3, MMP-9, IL-1, and TNF-*α* level in observation group presented depletion, suggesting that catgut embedding plus warm needle moxibustion can effectively reduce osteoarthritis in elderly patients.

Moreover, similar to control group, pain, knee joint function, and quality of life of patients in treatment group were also remarkably improved relative to those before treatment, but improvement in observation group was more marked. Though curative efficacy presented no difference between two groups, clinical cure proportion in observation group presented elevation relative to control group, suggesting that catgut embedding plus warm needle moxibustion in treating KOA may further optimize the curative efficacy and be more beneficial in pain relief and knee joint function and quality of life improvement.

However, the study had several limitations. First, the burials in the included studies may not be uniform, the method quality is poor, and confounding factors may be introduced. Second, the sample of our study was relatively small. All above limitations will be perfected in near future.

## 5. Conclusion

In conclusion, warm needle moxibustion plus functional exercise can effectively improve the clinical symptoms of KOA patients, and improve their knee joint function and inflammatory response, which is worthy of clinical reference.

## Figures and Tables

**Figure 1:** WOMAC scores and total scores of pain, stiffness, and daily activity difficulty in two groups before and after treatment. Note: ^∗^*P* < 0.05, vs. before treatment; # *P* < 0.05, vs. control group.

**Figure 2:** The levels of inflammatory cytokines in two groups before and after treatment. Note: ^∗^*P* < 0.05, vs. before treatment; # *P* < 0.05, vs. control group.

**Figure 3:** Quality of life in two groups. Note: ^∗^*P* < 0.05, vs. before treatment; # *P* < 0.05, vs. control group.

**Table 1:** Lequesne scores for osteoarthritis in two groups.

Groups	*N*	Before treatment	After treatment	*t*	*P*
Control group	60	14.26 ± 2.03	7.29 ± 2.37	9.28	< 0.001
Observation group	60	13.58 ± 1.98	4.59 ± 1.05	5.87	< 0.001
*t*		0.98	4.28		
*P*		0.631	0.016		

**Table 2:** Clinical efficacy in two groups.

Groups	*N*	Clinical cure	Markedly effective	Improved	Ineffective
Control group	60	38 (63.33)	14 (23.33)	6 (10.00)	2 (3.34)
Observation group	60	22 (36.67)	16 (26.66)	10 (16.67)	(20.00)

## Data Availability

Data generated in this study are available from the corresponding author under reasonable requests.
